The article "Flavonols and Flavones as Potential anti-Inflammatory, Antioxidant, and Antibacterial Compounds" was published in 2022. Journal: Oxid Med Cell Longev.

# Flavonols and Flavones as Potential anti-Inflammatory, Antioxidant, and Antibacterial Compounds

**DOI:** 10.1155/2022/9966750

**Published:** 2022-09-06

**Authors:** Maria do Socorro S. Chagas, Maria D. Behrens, Carla J. Moragas-Tellis, Gabriela X. M. Penedo, Adriana R. Silva, Cassiano F. Gonçalves-de-Albuquerque

**Affiliations:** ^1^Laboratório de Imunofarmacologia, Departamento de Bioquímica, Universidade Federal do Estado do Rio de Janeiro, Rio de Janeiro, RJ CEP 20211-010, Brazil; ^2^Programa de Pós-Graduação em Biologia Molecular e Celular (PPGBMC), Universidade Federal do Estado do Rio de Janeiro, Rio de Janeiro, RJ CEP 20211-010, Brazil; ^3^Programa de Pós-Graduação em Ciências e Biotecnologia (PPBI), Instituto de Biologia, Universidade Federal Fluminense, Niterói, RJ 24020-141, Brazil; ^4^Laboratório de Imunofarmacologia, Instituto Oswaldo Cruz, Fiocruz, Rio de Janeiro, RJ 21040-900, Brazil; ^5^Laboratório de Produtos Naturais para Saúde Pública (LPNSP), Instituto de Tecnologia em Fármacos – Farmanguinhos, Fiocruz, Rio de Janeiro, RJ 21041-000, Brazil; ^6^Programa de Pós-Graduação em Biologia Celular e Molecular (PPGBCM), Instituto Oswaldo Cruz, Fiocruz, Rio de Janeiro, RJ 21040-900, Brazil; ^7^Programa de Pós-Graduação em Neurociências (PPGNEURO), Instituto de Biologia, Universidade Federal Fluminense, Niterói, RJ 24020-141, Brazil

## Abstract

Plant preparations have been used to treat various diseases and discussed for centuries. Research has advanced to discover and identify the plant components with beneficial effects and reveal their underlying mechanisms. Flavonoids are phytoconstituents with anti-inflammatory, antimutagenic, anticarcinogenic, and antimicrobial properties. Herein, we listed and contextualized various aspects of the protective effects of the flavonols quercetin, isoquercetin, kaempferol, and myricetin and the flavones luteolin, apigenin, 3′,4′-dihydroxyflavone, baicalein, scutellarein, lucenin-2, vicenin-2, diosmetin, nobiletin, tangeretin, and 5-O-methyl-scutellarein. We presented their structural characteristics and subclasses, importance, occurrence, and food sources. The bioactive compounds present in our diet, such as fruits and vegetables, may affect the health and disease state. Therefore, we discussed the role of these compounds in inflammation, oxidative mechanisms, and bacterial metabolism; moreover, we discussed their synergism with antibiotics for better disease outcomes. Indiscriminate use of antibiotics allows the emergence of multidrug-resistant bacterial strains; thus, bioactive compounds may be used for adjuvant treatment of infectious diseases caused by resistant and opportunistic bacteria *via* direct and indirect mechanisms. We also focused on the reported mechanisms and intracellular targets of flavonols and flavones, which support their therapeutic role in inflammatory and infectious diseases.

## 1. Introduction

Flavonoids are an essential and diversified class of secondary plant metabolites present in different concentrations in the leaves, flowers, roots, and fruits. Flavonoid concentrations are influenced by natural factors such as temperature, ultraviolet (UV) radiation, season, pollutant, drought, and salinity stress owing to their effect on plant metabolism (Li [1]). The preparations containing flavonoids has been used to treat various human diseases. Flavonoids have anti-inflammatory, antimutagenic, anticarcinogenic, and antimicrobial properties [2–4]. They modulate the activities of several enzymes, including xanthine oxidase (XO), cyclooxygenase (COX), lipoxygenase (LOX), and phosphoinositide 3-kinase [5]) involved in pathological processes.

Inflammation is a complex biological response to noxious stimuli. It protects organisms against pathogens, cell damage, and irritating chemicals. Moreover, it initiates the healing process, which involves different cells and chemical mediators [6, 7]. Nevertheless, exacerbated and uncontrolled inflammation can also cause deleterious tissue damage. Flavonoids can alter cellular responses and production of chemical mediators related to inflammatory processes [8] caused by many agents, including natural toxins, pharmaceuticals, heavy metals, and environmental chemicals [9].

Oxidative stress is induced by mitochondrial dysfunction and inflammation [10, 11]. Continuous oxidative stress generates reactive oxygen species (ROS) and reactive nitrogen species (RNS), causing lipid peroxidation, protein and nucleic acid oxidation, and even cell death [12]. These effects are dependent on redox balance because they act as damaging agents and physiological regulators of cell functions [13]. Plant extracts are valuable sources of bioactive compounds with antioxidant properties. For example, honey shows antioxidant and anti-inflammatory properties owing to its high flavonoid content [14–16]. Moreover, honey intake led to reduction in malondialdehyde and ROS levels generated by high physical activity in athletes and murine models [17–20]. A recent review discussed the role of consuming plant foods rich in antioxidants in protection against cognitive decline [12].

Similar to all secondary plant metabolites, plant defense mechanisms include flavonoid production; for example, a plant under attack by microorganisms may trigger the production of flavonoids having antimicrobial effects [21]. Herein, we discussed many aspects of the protective effects of flavonols and flavones in detail.

## 2. Flavonoids: Structural Characteristics and Subclasses

Flavonoids present a C6-C3-C6 carbon skeleton structure that consists of at least two aromatic rings, called A and B, linked by the three carbons chain that can form a heterocyclic ring containing oxygen (ring C) with ring A (Figure 1) [175]. Flavonoids are divided into flavones, flavonols, flavanones, flavanols, isoflavones, leucoanthocyanidins, anthocyanidins, and chalcones [5] (Figure 2). The subclasses are determined by minor structural variations, including the absence of ring C, position of the bond between ring B and ring C, degree of unsaturation, and ring C oxidation [22, 23]. In addition, substitutions at these rings can lead to differences in hydrogenation, hydroxylation, methylation, malonylation, sulfation, and glycosylation, which determine different pharmacological activities [5]. Currently, there have been reported more than 9000 different flavonoids [24].

We focused on two groups: (a) flavones that have a double bond between C2 and C3 in the flavonoid skeleton, without substitution at C3 and oxidized at C4, and (b) flavonols that differ from flavones by a hydroxyl group at C3 (Figure 2).

### 2.1. Flavonols and Flavones: Importance, Occurrence, and Food Sources

Almost all natural flavonoids exist in plants in O-glycosides or C-glycosides forms. C-glycosides are sugar moieties combined directly to flavonoid backbone as C–C covalent bonds. O-glycosides are formed by attaching sugar to hydroxyl oxygen [25]. The most common sugars attached to these flavonoids are D-glucose and L-rhamnose, but at least eight monosaccharides or combinations thereof may bind to different hydroxyl groups of flavonoids, resulting in a large number of known glycosides [26, 27]. They are widely present in plants and are potential metabolites involved in plant signaling and defense mechanism. Furthermore, they are vital ingredients in human diet and have significant health benefits [28–30]. Flavonols, which are primary flavonoids in nature, are found in various fruits and vegetables, such as apples, berries, grapes, tomatoes, and onions, and play a key role in attracting pollinators and seed disseminators [27, 31].

Flavones and flavonols have antioxidant effects and are essential for protecting plants from UV radiation [32, 33]. Quercetin (3,3′,4′,5,7-pentahydroxyflavone) is one of the most representative flavonoids, widely distributed in nature, and an abundant dietary flavonol, found in food, such as onions, peas, and apples [22, 26]. Quercetin-3-O-rutinoside, known as rutin (3,3′,4′,5,7-pentahydroxyflavone-3-rhamnoglucoside) and also called vitamin P due to contribute to reducing the permeability of blood vessels, was introduced in the market and has been explored for important pharmacological effects [34]. Luteolin (*3*′,*4*′,*5*,*7*-tetrahydroxyflavone) and apigenin (*4*′,*5*,*7*-trihydroxyflavone) are the main flavones found in food, such as onions, celery, red pepper, and grapes, and have a wide range of effects in biological systems, including anti-inflammatory and anticarcinogenic [35]. Luteolin is found in cereals and herbs, and glycosylated luteolin in vegetables such as carrots and broccoli [31, 36]. Luteolin inhibits cancer in head and neck squamous cell carcinoma (HNSCC) xenograft in a mouse model by inhibiting p300 lysine acetyltransferase activity *via* acting at multiple levels of gene expression, miRNA expression, and miRNA processing [37]. Luteolin effectively prevented pulmonary and hepatic fibrosis [38, 39] and reduced cancer cell proliferation [40]. Both effects are due to the reduction in oxidative stress and inflammatory responses [41]. Interestingly, luteolin can also play a protective role in inflammation and cancer by modulating the microbiota ([42]. The flavonoid hesperidin possesses antioxidant and anti-inflammatory properties and plays a role in inhibition of tumor cell metastasis and angiogenesis [43].  Table 1 shows some flavones and flavonols aglycones and its natural sources and content (mg/100 g or mg/100 ml).

### 2.2. Inflammation

Inflammation is a complex response initiated by an insult by chemical, physical, or biological agents, which leads to resolution and promotes tissue repair [54, 55]. During the inflammatory process, immune system cells, such as neutrophils, monocytes, eosinophils, and lymphocytes, migrate to the lesion site [56, 57].

The lipid mediators eicosanoids and cytokines produced during the inflammatory response cause vascular and cellular alterations such as vasodilation, an increase in vascular permeability and activation, adhesion, and cellular transmigration [54]. The increase in the concentrations of inflammatory cytokines, such as interleukin (IL)-1*β* and tumor necrosis factor (TNF)-*α*, is crucial for leukocyte migration to the lesion [58–60]. The production of mediators and increased vascular permeability generate an exudate rich in plasma proteins [61]. The production of inflammatory mediators leads to endothelial increased permeability and leukocyte activation and migration to the injury site, cellular, and tissue damage and triggers the characteristic symptoms of inflammation, known by the five cardinal signs: pain, redness, heat, edema, and loss of function [54, 62]. When leukocytes reach the inflammation site, they are activated and respond to eliminate noxious stimuli, thus releasing the content of their toxic granules, which includes ROS, reactive nitrogen species (RNS), proteinase, cathepsin G, and elastase [61, 63].

The inflammatory process involves the production of numerous cytokines that bind to cellular receptors triggering intracellular signaling, such as JAK kinase, phosphatidylinositol-3-kinase (PI3K), V-Akt murine thymoma viral oncogene homolog 1 (AKT1), inhibitory kappa B kinase (IKK), and mitogen-activated protein kinases (MAPKs), which are responsible for the activation and nuclear translocation of transcriptional factors (signal transducer and activator of transcription [STAT], nuclear factor kappa B [NF-*κ*B], and activator protein 1[AP-1]) [64–67].

Inflammatory responses must be fine-tuned because if exacerbated, it will damage tissues and, if insufficient, will not cause complete elimination of pathogens. Exacerbation of immune response with uncontrolled inflammation results in poor outcomes [68]. Drugs or natural compounds with strong anti-inflammatory effects allow microbes to grow and decrease survival [69]. However, adequate anti-inflammatory effects may prevent organ damage and improve host survival [69, 70].

### 2.3. ROS and Oxidative Stress

ROS are presented by one or more unpaired electrons produced in cells during mitochondrial oxidative metabolism and in cellular response to xenobiotics, cytokines, bacterial invasion, UV radiation, and pollutants, collectively known as oxidizing agents [71]; they promote cascade reactions and cause oxidative damage [71, 72].

Normal metabolism generates reactive species that play a prominent role in physiological functions, including gene expression, cell signaling, and immune responses. Antioxidants neutralize reactive species in excess [71, 72]. An antioxidant is a molecule able to donate an electron to a rampaging free radical and neutralize it [73]. Some antioxidants can interact with other antioxidants regenerating their original properties called the “antioxidant network” [74]. They neutralize ROS by different mechanisms including directly scavenging free radicals, directly scavenging free radicals, and inhibiting lipid peroxidation between others [75]. Antioxidant system can be enzymatic or nonenzymatic. The nonenzymatic system blocks the initiation of oxidation. The enzymatic system comprises antioxidant enzymes such as superoxide dismutase (SOD), catalase (CAT), glutathione peroxidase (GPx), and glutathione reductase (GR). In the nonenzymatic antioxidant system, glutathione (GSH); ascorbate (AsA); numerous simple phenolic acids such as hydroxybenzoic acids, hydroxycinnamic acids, and different flavonoid compounds; carotenoids such as xanthophylls, beta-carotene, and *α*-carotene; vitamin E; and pigments such as chlorophylls, betaxanthins, betalains, and betacyanins such as amaranthine, isoamaranthine, betanidine, and isobetadine are the most noticeable components ([76]). Antioxidants act by stabilizing ROS. An imbalance in ROS production and antioxidant activity in biological systems causes oxidative stress. As a result of this imbalance, cellular dysfunction may occur *via* modulating gene expression, protein stability, and membrane fluidity, leading to cell damage and death [72]. An increase in reactive species levels occurs with aging and the development of diseases, including cancer, Parkinson's disease, diabetes, and cardiovascular diseases [77]. ROS increase is linked to different diseases, reviewed by [78]. For instance, excessive ROS accumulation leads to glutathionylation modification and proteasomal degradation of MAP kinase phosphatase-1, which prevents insulin signaling. Also, ROS in excess inactivates AKT, inhibiting glucose uptake, which eventually causes type 2 diabetes. In addition, mitochondria-derived ROS elicit the production of NLRP3 and IL-1*β*, accounting for an inflammatory phenotype in atherosclerosis pathogenesis. Furthermore, phosphorylated tau protein and A*β* are risk factors in Alzheimer's disease, which originate from the downregulated Nrf2 and increased ROS burden. Finally, extracellular and intracellular ROS activate TGF-*β* signaling triggering the epithelial-mesenchymal transition of epithelial cells and survival of circulating tumor cells during cancer metastasis [78].

The search for new antioxidant compounds as therapeutic agents for diseases associated with imbalance in reactive species production and clearance is gaining attraction of researchers. Natural antioxidants, such as phenolic compounds (flavonoids and phenolic acids), have emerged as primary therapeutic agents as nonenzymatic antioxidants because they can sequester ROS [79]. They also act as anti-inflammatory agents.

### 2.4. Limitations Associated with the Use of Flavonoids

We consume fruits and vegetables that containing flavonoids, such as apples, berries, onions, and broccoli, on a daily basis [80, 81]. However, their bioavailability can vary. A trial conducted with 97 humans showed that the plasma concentrations of total polyphenolic metabolites was 0–4 *μ*mol/L after an intake of 50 mg aglycone equivalents, and the urinary excretion was 0.3–43% of the ingested dose [82]. Flavonoids are absorbed in the small intestine. Flavonoids that cannot be absorbed in the small intestine are degraded in the colon by microorganisms to phenolic acids [83].

The absorption of flavonoids from food was long considered to be very low, as they are present in foods linked to sugars such as *β*-glycosides (except catechins). Only aglycones forms were considered able to pass the gut wall, and no enzymes that can split these predominantly *β*-glycosidic bonds are secreted into the gut or present in the intestinal wall [84]. Unlike terpenes with high bioavailability, flavonoids can have low bioavailability due to the extensive first-pass effect and glucuronidation [85]. However, research on the mechanisms for aglycone transfer across the gut wall is lacking. In a study on ileostomized humans, the absorption of orally administered quercetin was 24%. These data show that humans absorb appreciable amounts of quercetin and that absorption of glycosides in the small intestine is possible. Humans consume, on average, between 0.45 and 1.17 mg of apigenin daily [86]. Apigenin when taken orally (whose bioavailability is about 30%) is systemically absorbed and recirculated by enterohepatic and local intestinal pathways [87].

Despite these concerns about bioavailability, which seems to be influenced by their chemical nature, flavonoids effectively prevent or improve diseases. There are three possible explanations for this: (1) act in the lumen or intestinal epithelium, (2) act in the peripheral tissues even at very low circulating levels, or (3) the microbial metabolites of flavonoids are also active in the peripheral tissues [88]. Flavonoid amount consumed through food is generally nontoxic. However, when consumed in large amount, they can show toxic effects. Administration of high doses (≥200 mg/kg) and prolonged use of luteolin may increase hepatic enzyme activity; however, no significant liver damage was observed, whereas low doses (≤50 mg/kg) are hepatoprotective [89].

The purification or production of bioactive compounds on a large scale is challenging. Although a specific bioactive compound has been identified and proven to be beneficial in treating inflammatory or infectious diseases, its purification or bioengineering remains a challenge. Moreover, where bioactive flavonols have been identified in natural food, the among ingested is difficult to determine because it varies from place to place depending on the environment in which the plant grows. Another crucial challenge is the development of optimum delivery formulations. Nevertheless, the flavonoid properties in biological systems are indisputable because they are bioactive compounds with the potential to treat or prevent diseases; therefore, future studies based on better delivery systems, such as nanoformulations, should be encouraged [90, 91].

### 2.5. Flavonols and Inflammation

The current strategies for treating inflammatory and infectious diseases often present side effects that markedly affect the quality of life of patients. In addition, the use of immunosuppressants may be essential to control the immune response in infectious diseases; however, it can increase the risk of spread of the infection and should be used with caution. Flavonols, such as quercetin, kaempferol, and myricetin, are the most common plant flavonoids. We discussed recent studies on anti-inflammatory effects of flavonols and listed them in Table 1.

### 2.6. Anti-Inflammatory Effects of Quercetin, Isoquercetin, Kaempferol, and Myricetin

First isolated in 1857 from oak (*Quercus*), quercetin is probably the most investigated flavonoid. It has strong and prolonged anti-inflammatory effects [75, 92, 93]. Quercetin acts through several mechanisms such as by inhibiting lipopolysaccharide (LPS)-induced TNF-*α* production in macrophages [94], inhibiting LPS-induced IL-8 in A549 lung carcinoma epithelial cells [95], and inhibiting the production of inflammatory mediator-producing enzymes such as COX and LOX [96, 97]. Quercetin showed cardioprotective effect against isoproterenol-induced myocardial infarction in rats [98] (Figure 3). Additionally, it reduced levels of biomarkers of ischemic induction, such as creatine kinase myocardial band (CK-MB) and cardiac troponin I (cTnl), inhibited inflammatory cell infiltration into the myocardium, reduced the expression of TNF-*α* and IL-6, and inhibited upregulation of calpain genes 1 and 2 that protect the myocardium [98].

Treatment with quercetin improved LPS-induced inflammatory damage in pulmonary fibroblasts by increasing cell viability, Treatment with quercetin improvedaverting apoptosis, and reducing pro-inflammatory cytokine production (TNF-*α* and IL-6) [95]. In an experimental model of acetic acid-induced gastric ulcers in rats, quercetin, isolated from *Madhuca indica*, inhibited cytokines (IL-1*β* and TNF-*α*), NO, and prostaglandin production by downregulating COX-2 expression [99]. Similarly, quercetin treatment reduced IL-1*β* and TNF-*α* levels [100]. Macrophage inflammatory protein 1*α*/chemokine (C-C motif) ligand 3 (MIP-1*α*/CCL3) is a key to monocytes/macrophage recruitment, and the release from adipocytes and macrophages tissue causes tissue inflammation [101]. Quercetin suppressed MIP-1*α* effects by downregulation of CCR1/CCR5 and inhibition of activation of c-Jun N-terminal kinase (JNK), p38 mitogen-activated-protein kinase (MAPK), and IKK and I*κ*B*α* degradation [3].

Oral administration of quercetin for the treatment of arthritis induced by inactive *Mycobacterium butyricum* in a rat model showed that quercetin could diminish inflammatory markers, such as IL-1*β*, C-reactive protein, and MPC-1 and restore the plasma antioxidant capacity. In addition, it inhibited 12/15-LOX activity in the lungs and liver and increased heme oxygenase-1 (HO-1) expression in joints and lungs [102]. Quercetin treatment decreased inflammation and attenuated pathological alterations in the pancreas and ileum of animals with acute necrotizing pancreatitis. This suggests that the flavonoid acts by partial inhibition of TLR4/MyD88/P38 and MAPK ERK, thus reducing inflammation and interrupting intestinal damage [103]. In a model of monohydrate crystal–induced arthritis fatty acids activates TLR2 inducing interleukin-1*β* production via the ASC/caspase 1 pathway [104]. In addition, quercetin inhibited the release of ROS, IL-1*β*, and IL-18, resulting in the protection of mitochondrial integrity in Caco-2 cells stimulated with *Escherichia coli* [105]. It also blocked the inflammasome NLRP3 activation in the rat kidneys [106, 107].

Moreover, quercetin suppressed the CXCR4 upregulation in otitis media induced by non-typificable gram-negative bacillus *Haemophilus influenzae* (NTHi), both *in vitro* and *in vivo* [102]. It downregulated the TLR3/Myd88 signaling by blocking NF-*κ*B activation [108] and IKK*α* and p38 phosphorylation in mice inoculated with NTHi [102]. A recent study showed that isoquercetin treatment reversed weight loss, decreased glucose levels, and increased insulin production in streptozotocin-induced diabetic rats. Furthermore, isoquercetin reduced lipid peroxidation by increasing SOD and CAT activity, which improved the lipid profile in the diabetic group. In addition, this flavonol suppressed inflammatory genes that code for NF-*κ*B, IL-1, IL-6, TLR, TNF-*α*, and COX-2 [109].

Kaempferol (from genus *Kaempferia*) is a flavonol abundantly present in various species and plant-derived foods; it has been shown to inhibit adipogenesis by blocking 3 T3-L1 differentiation and lipid accumulation in mature adipocytes. It modulated adipogenic gene expression and decreased lipid accumulation in mature adipocytes (CEBPA) *via* upregulating mRNA expression of Pnpla2 and Lipe [110]. Similarly, kaempferol treatment reduced lipid and protein accumulation along with the expression of the adipogenic markers PPAR*γ* and C/EBP*α* in 3 T3-L1 cells [108]. These changes in adipocyte lipid metabolism affect the response of adipocytes to the production of inflammatory mediators.

First isolated from the bark of *Myrica nagi*, myricetin is a common flavonol occurring also in both free or glycosylated forms, with anti-inflammatory activity and cardioprotective effect, which prevents myocarditis by reducing apoptosis [111]. It markedly reduced cleaved caspase-3 and Bcl-2 levels and increased Bax levels in H9c2 cells. The flavonol decreased MCP-1 and I*κ*B*α* phosphorylation levels by blocking the NF-*κ*B activation in LPS-challenged H9c2 cells. Treatment with semisynthetic flavone derived from myricetin (the M10 compound) prevented chronic inflammation and ulcerative colitis induced by azoxymethane/dextran in colorectal tumorigenesis [24].

### 2.7. Flavones and Inflammation

Flavones are characterized by the absence of a hydroxyl group at C3 when compared to flavonol that also exhibit structural variations of hydroxylation, O-methylation, C-methylation, or prenylation. This wide range of structural combinations results in several types of flavones, making them as an abundant subclass [112]. Herein, we discussed the most frequent flavones present in human diet, luteolin, and apigenin. Luteolin modulates the immune response more efficiently than other naturally derived compounds such as quercetin, genistein, and hesperidin [113] (Table 2). Besides, apigenin is also known for its anti-inflammatory and antioxidant effects by inhibiting cytokine secretion and downregulating enzymes such as inducible nitric oxide synthase (iNOS) and COX-2 [114].

### 2.8. Luteolin, Apigenin, and Inflammation

Luteolin and apigenin are the most abundant flavones occurring in nature. They differ structurally by the presence of a hydroxyl group at C3` (Figure 4).

Luteolin was first isolated in 1829 as the main yellow-colored compound extracted from *Reseda luteola* and structure confirmed by synthesis in 1900 [115]. Luteolin has antimicrobial, anti-inflammatory, chemopreventive, chemotherapeutic, cardioprotective, antidiabetic, neuroprotective, and antiallergic properties [116–119]. Moreover, consumption of luteolin-rich food reduces the risk of developing chronic diseases [120].

Luteolin exhibited its anti-inflammatory effect by reducing the production of pro-inflammatory agents, such as NO, prostaglandin E2 (PGE2), TNF-*α*, MMP-2, MMP-8, and MMP-9, and by downregulating COX-2, iNOS, MMP-3, and MMP-13 expression in both *in vitro* and *in vivo* arthritis models [1, 113]. Luteolin also showed effects in human neutrophils by inhibiting NET formation, elastase release, CD11 expression, chemotaxis, and the RAF1-MEK-1-Erk signaling pathway, resulting in decreased neutrophil infiltration and activation, thereby attenuating the inflammatory response [1]. It also blocked ROS, TNF-*α*, IL-6, and nitric oxide (NO) production in human and mouse cells [121].

In addition, luteolin showed a cardioprotective effect in cardiomyocyte cultures and experimental type 1 diabetes. This flavone reduced inflammation by inhibiting the NF-*κ*B signaling, cytokine production, and oxidative stress by blocking the activation of the nuclear factor 2 (NRF2) pathway. It has also been shown to prevent cardiac fibrosis, hypertrophy, and dysfunction in diabetic rats [122]. Moreover, luteolin inhibited the production of IL-8 and COX-2 and reduced the expression of iNOS and NO in colon HT-29 cells [123]. Hence, it has emerged as a potential candidate for the treatment of bowel disease because of its ability to modulate intracellular inflammatory signaling cascade. Inhibition of the JAK/STAT signaling pathway seems to be a key mechanism for anti-inflammatory action of luteolin in bowel diseases [124]. These results indicate that luteolin negatively modulates the main signaling pathways involved in the intestinal inflammation.

Luteolin inhibited the expression of TNF-*α*, IL-1*β*, and IL-6; suppressed I*κ*B*α* and NF-*κ*B p65 phosphorylation levels; and downregulated the expression of MMP-2 and MMP-9 in *S. aureus*-induced mastitis [125], showing its potential in reducing tissue damage and inflammation caused by *S. aureus*-induced mastitis. Moreover, luteolin showed effects in arthritis models through the involvement of metalloproteinase [113]. Luteolin plays a critical role as an anti-inflammatory agent by reducing the production of inflammatory mediators, inhibiting crucial inflammatory intracellular pathways, and blocking the translocation and activation of inflammatory transcription factors. Therefore, it is a potential agent for the treatment and prevention of inflammatory, infectious, and metabolic diseases.

Apigenin, a constituent from celery (*Apium graveolens*) also common in other food plants, such as parsley and chamomile [49], has therapeutic potential for various diseases (diabetes, cancer, and neurological and cardiovascular disorders) [126], considering its anti-inflammatory, antioxidant, and anticancer effects. The mechanism of action of apigenin involved the suppression of p65 phosphorylation in monocytes and macrophages and reduction in the expression of COX-2 and NO in rat macrophages [8]. Zhang et al. have reported that apigenin inhibited CD38, an inflammatory biomarker, reduced pro-inflammatory cytokines, and led to reduction in adipose tissue mass in a metabolic syndrome model [127]. Treatment with apigenin prevented pulmonary fibrosis and bleomycin-induced inflammation by decreasing TNF-*α* and TGF-*β*1 levels and attenuating the reduction in SOD activity [128]. An *in vivo* experiment on concanavalin A-stimulated rat splenocytes showed that apigenin prevented iNOS induction, downregulated COX-2 expression, and reduced pro-inflammatory cytokine production (TNF-*α*, IFN-*γ*, and IL-2). The flavone has also demonstrated an antiproliferative effect on lymphocytes [114].

### 2.9. Effect of Other Flavones on Inflammation

Other flavones with anti-inflammatory effects, such as 3′,4′-dihydroxyflavone, baicalein, scutellarein, lucenin-2, vicenin-2, diosmetin, nobiletin, tangeretin, and 5-O-methyl-scutellarein, have been described (Figure 5).

3′,4′-Dihydroxyflavone suppressed the MAPK and NF-*κ*B signaling pathways, in addition to the inhibition of NO, PGE2, and pro-inflammatory cytokine production in microglial cells and mice [129]. Baicalein, one of the main constituents of *Scutellaria baicalensis* Georgi [127] improved motor deficit and attenuated brain injury in rats chronically exposed to rotenone. Baicalein inhibited IL-6, TNF-*α*, and NO production, blocked I*κ*B*α* phosphorylation and NF-*κ*B translocation, and negatively modulated TLR4 in BV2 microglial cells. Similarly, scutellarein (*Scutellaria barbata*) improved LPS-induced cognitive deficit in rats and decreased the levels of hippocampal malondialdehyde (MDA) and antioxidant defense elements such as SOD, catalase, and GSH [130]. Thus, the authors suggest possible mechanisms underlying anti-inflammatory activity as inhibition of the levels of NF-*κ*B, TNF-*α*, IL-6, and NRF2, in addition to the inhibition of autophagy markers and decreased expression of matrix metalloproteinase.

Diosmetin (3′,5,7-trihydroxy-4′-methoxyflavone) is a flavone common in *Citrus* species, which exerts anti-inflammatory and other effects [131]. Diosmetin-7-O-rutinoside, known as diosmin (3′,5,7-trihydroxy-4′-methoxyflavone 7-rhamnosylglucoside), is well stablished to treat vessel permeability and inflammatory diseases. A recent study was showed that diosmetin attenuates experimental ulcerative colitis in rats via suppression of NF-*κ*B, TNF-*α*, and IL-6 signaling pathways correlated with downregulation of apoptotic events [132].

Glycosylated flavones, lucenin-2, vicenin-2, and scutellarein-2, obtained from *Korthalsella japonica*, possess anti-inflammatory activity [133]. Both the extract and isolated flavones inhibited the production of NO and reduced the expression of iNOS and COX-2 in LPS-stimulated RAW 264 cells (M. K. [133]). Vicenin-2 negatively regulated the secretion of cytokines (TNF-*α* and IL-1*β*) and increased the expression of IL-10 and IL-1Ra in LPS-induced mononuclear cells [134]. Furthermore, vicenin-2 inhibited the reporter activity of NF-*κ*B and increased homodimerization of P50 subunit of transcription factor by heterodimerization of P50/P65 [135].

Nobiletin, a polymethoxyflavone (3′,4′,5,6,7,8-hexamethoxyflavone), reduced the myeloperoxidase activity in the pancreas, cellular damage, and phosphorylation of p38 and AKT in a model of acute peritonitis. It also reduced the levels of TNF-*α*, IL-1*β*, IL-6, and IL-10, attributing to its anti-inflammatory activity [136].

Tangeretin, a flavone isolated from dried fruit shells of *Citrus tachibana*, attenuated colitis parameters such as colon shortening; activation of myeloperoxidase, NF-*κ*B, and MAPKs; production of IFN-*γ*, TNF-*α*, and IL-17; and expression of COX-2 and iNOS. Therefore, it has shown significant anti-inflammatory effect [137]. Hydroethanolic extract of *Arrabidaea chica* leaves and its isolated flavone 4′,6,7-tri-hydroxy-5-methoxyflavone (5-O-methyl-scutellarein) dose-dependently inhibited inflammatory cell recruitment and TNF-*α*, IL-1*β*, and IL-10 production [138].

A recent study reviewed preclinical and clinical data on anti-inflammatory and analgesic properties of flavonoids; most data demonstrated the potential therapeutic role and efficacy of flavonoids in cardiovascular diseases, osteoarthritis, Parkinson's disease, colitis, cancer pain, arthritis, and neuropathic pain. Nevertheless, the mechanisms of action of flavonoids have yet to be fully elucidated. Considering the pharmacological activities of flavonoids, it would be promising to further develop delivery formulations containing flavonoids to treat inflammatory diseases and pain [139].

Different approaches to evaluate the anti-inflammatory activity of flavones described above, both *in vitro* and *in vivo*, showed a reduction in the production of pro-inflammatory mediator, and inhibition of activation of the signaling pathway and nuclear factor. Regardless of the chosen model of arthritis, colitis, or gastric ulcer, flavones inhibited different signaling pathways, production of mediators, transcription factor activation, and ROS production.

### 2.10. Antioxidant Effects of Flavonols and Flavones

The balance between ROS production and antioxidant cell mechanisms regulates oxidative stress in cells and can lead to cell damage when unregulated. Antioxidant enzymes, SOD and CAT, can directly detoxify the generated ROS or facilitate antioxidant activity using GSH as a reducing agent [143]. CAT is responsible for peroxide decomposition in a cell [144].

The antioxidant activity of quercetin can be explained by its direct effect on GSH, signal transduction pathways, enzymatic activity, and ROS, which maintain oxidative balance. Quercetin regulates the levels of GSH, a hydrogen donor in decomposition of H_2_O_2_ to H_2_O, by inducing its synthesis. By influencing the signal transduction pathways, the compound can inhibit the enzymatic activity of numerous enzymes associated with oxidative mechanisms, such as acetylcholinesterase (AChE) and butyrylcholinesterase (BChE), and enhance the expression levels of antioxidant enzymes such as SOD, CAT, and GSH peroxidase. Finally, quercetin can remove ROS through various mechanisms involved in regulation of ROS production and modulation of antioxidant-related gene expression. Clinically, quercetin exhibits antitumor effect and is used for cancer and metastasis prevention [145]. It has also been shown to have therapeutic effects in cardiovascular diseases and significant antidepressant outcome [146]. Quercetin isolated from *Flaveria bidentis* (L.) inhibited ROS production in human mononuclear cells and polymorphic leukocytes more efficiently than that of vitamin C [147]. Quercetin reversed the oxidative damage induced by FeSO_4_ ferrous ions in bovine sperm cells [148]. The flavonol also induced the expression of HO-1 and the subsequent end product, suppressing oxidative stress derived from NADPH oxidase [142]. Furthermore, quercetin decreased MDA levels in the myocardial tissue and activated SOD and GPx enzymes [98, 142], demonstrating the antioxidant activity of quercetin in a rat model of myocardial infarction. In a similar study, treatment with quercetin decreased MDA levels in the myocardial tissue and further stimulated SOD and GPx enzymes [149].

Luteolin attenuated oxidative damage and reduced the generation of intracellular ROS by inducing the expression of the antioxidant enzyme HO-1, thus counteracting the damage induced by H_2_O_2_ in rat cortical primary cell cultures [141]. Treatment with the flavone normalized AST and ALT levels. The protective role of luteolin against ROS and oxidative damage occurs by normal GSH level restoration and lipoperoxidation suppression in the plasma and liver tissues [140]. Moreover, the flavone blocked superoxide anion and ROS production in human neutrophils [150], strengthening the role of luteolin as an antioxidant agent. Chanput et al. evaluated the antioxidant activity of three classes of flavonoids: (i) flavonol: quercetin and myricetin; (ii) flavanone: eriodictyol and naringenin; and (iii) flavone: luteolin and apigenin [151]. The flavonol group (myricetin and quercetin) showed the best antioxidant activity among the three groups, which might be due to the presence of more hydroxyl groups in their structure and the presence of double bond between C2 and C3 of the aromatic ring that improve their antioxidant properties by the electron distribution pattern [152] compared to the other groups.

### 2.11. Antibacterial Activity of Flavones and Flavonols

Several studies have supported the use of medicinal plants for their antimicrobial activities. Flavonoids act on different microorganisms. Herein, we discuss their effects on resistant and opportunistic bacteria. Antibiotic abuse may lead to the select bacterial resistance to current drugs. Medicinal plant extracts contain a variety of phytochemical substances that can act synergistically to inhibit the bacterial growth and prevent the development of drug resistance.  Table 3 shows the flavonoids used for antibacterial purposes and their mechanisms of action.

Methanolic fraction of the extract from *Justicia wynaadensis* contains 3,3,4-trihydroxyflavone that exhibits antimicrobial activity against multiresistant and opportunistic organisms. Flavones can effectively kill bacteria present in diabetic wounds such as *Enterococcus faecalis*, *Streptococcus aureus*, *Klebsiella pneumoniae*, *Enterobacter aerogenes*, *Escherichia coli*, and *Pseudomonas aeruginosa* [153]. The methanolic extract of *J. wynaadensis* also showed antibacterial activity against *K. pneumoniae* (Ponnamma SU2015). The methanolic extract of *Tragia involucrata* was effective against *Enterobacter aerogenes*, *P. aeruginosa*, *S. aureus*, *Proteus vulgaris*, and *E. coli* associated with diabetic foot ulcer and ICU [154].

The methanolic root extract from *Garcinia macrophylla* is an important medicinal herb used to treat diverse diseases and disorders in Traditional Chinese Medicine and showed antimicrobial activity against bacterial strains of *Micrococcus luteus*, *E. faecalis*, *S. aureus*, *Staphylococcus epidermidis*, *Streptococcus uberis*, *P. aeruginosa*, *E. coli*, and *K. pneumoniae* isolated from burn wounds, with the lowest minimum inhibitory concentration against *S. epidermidis* and the highest MIC value against *E. coli* [150]. The authors observed equivalent values for minimum bactericidal concentration (MBC). The antibacterial activity of *Gentiana kurroo* methanolic extract overcame the results presented by other comparable studies [155].

The methanolic extract of *B. purpurascens* leaves, a medicinal herb containing diverse flavonoids (bergenin, catechin, naringenin, and myricetin), is used to treat wounds and bacterial infections. The extract exhibited strong antibacterial properties, particularly against *S. aureus* and *Streptococcus* spp. These results corroborate those of previous studies demonstrating the inhibition of growth of different bacteria by *Bergenia* spp. [156, 157] and that silver-plated nanoparticles from *Bergenia cilita* crude extract had antimicrobial activity against several bacterial strains. Moreover, *B. purpurascens* extract reduced the mortality caused by infection of mice with *S. aureus in vivo* [158, 159].

Microorganisms' growth and survival are associated with biofilm formation. Quorum sensing (QS) is an intercellular signaling or cell-cell communication process that is necessary for coordinating biofilm formation. The QS system is related to opportunism and resistance mechanisms developed by many bacterial strains. Blocking QS in bacteria is a far-reaching strategy for attenuating their virulence and making them more susceptible to elimination by the host immune system at lower doses of antibiotics. The modulatory effect of kaempferol-loaded chitosan nanoparticles on autoinducer (AI)-mediated anti-QS activity by *Chromobacterium violaceum* CV026 was used to evaluate the effect of this flavonol. Changes in bacterial cell density led to AI production *via* signaling molecules involved in communication among bacteria, composing QS, and managing growth. The results of anti-QS evaluation using the disk diffusion method showed that kaempferol produces a remarkable anti-QS effect; thus, its use against resistant bacteria is promising [158, 159].

Baicalin, a flavonol extracted from the Chinese medicinal plant *Scutellaria baicalensis*, has also demonstrated *in vitro* and *in vivo* anti-QS activities [160]. Baicalin concentrations below the MIC (sub-MIC) inhibited Pseudomonas biofilm formation, which increased the bactericidal effects of various conventional antibiotics. MIC and broth microdilution methods were used to evaluate the MIC and MBC of baicalin and antibiotics, biofilm inhibition assay, biofilm dispersion evaluation, and combined antibiotic use. Treatment with different concentrations of baicalin inhibited *P. aeruginosa* biofilm formation in a dose-dependent manner. The lower number of viable cells and lower biomass indicated a synergistic effect compared to treatment with flavonol alone and antibiotics [161], demonstrating that baicalin co-treatment increased the antimicrobial activities of three different antibiotics.

Treatment with sub-MIC of baicalein reduced QS. It decreased most virulence factors, corroborating previously reported data and demonstrating that baicalin exerts anti-QS activity against *P. aeruginosa* PAO1 by inhibiting the QS gene expression and production of signaling molecules such as acyl-homoserine lactone (AHL). Treatment with a sub-MIC of baicalin also considerably increased the survival rate of *C. elegans*. Moreover, baicalin inhibited the motility and production of the QS molecule pyocyanin and significantly reduced the number of colony-forming units (CFUs) of *P. aeruginosa* in implants [160]. Previous studies have also demonstrated reduced bacterial growth in implants treated with baicalin and antibiotics, particularly levofloxacin, ampicillin/clavulanic acid, and ceftazidime [162]). *In vivo* experiments have shown a higher survival rate of worms in the baicalin-treated group, which indicates that treatment with baicalin reduced the pathogenicity of *P. aeruginosa* in *C. elegans*. In addition, baicalin treatment increased the clearance of *P. aeruginosa* from the implants of infected animals in a peritoneal implant infection model.

Quercetin, both free and chitosan-associated, and baicalein have shown a potential inhibitory effect on biofilm formation, QS formation, and cytotoxicity in free mammalian cells treated with chitosan-based nanocapsules [163]. A transformed *E. coli* Top 10 biosensor strain showed QS formation. These results are in line with the data of a previous study [164] that suggested that these phytochemicals may inhibit biofilm formation [163]. Indeed, baicalin inhibited *P. aeruginosa* PAO1 biofilm formation, whereas quercetin showed the highest anti-QS effect in PAO1 strain [165].

The flavonol rutin inhibited QS, biofilm formation, and virulence genes in pathogenic *E. coli* APEC-O78 *in vitro*. Bioluminescence assay demonstrated that AI-2 secretion and activity were significantly decreased after rutin treatment, resulting in marked inhibition of biofilm formation. The expression of APEC virulence genes (csgA, csgB, Flic, FyuA, IucD, LsrB, LsrK, Rpos, H-NS, Luxs, and Pf) decreased after treatment with rutin. These results highlight the role of rutin in controlling *E. coli* pathogenicity. Furthermore, flavonols reduced cellular damage in type II pneumocytes infected with pathogenic *E. coli* by interfering with the QS, thereby inducing a decrease in AI-2 production, biofilm formation, and virulence gene expression [162].

The efflux pump proteins encoded by genes involved in bacterial cellular functions may cause antibiotic resistance. Crude extracts and 3′,4′,7-trihydroxyflavone compound extracted from *Myristica fragrans* Houtt. (MSF) have shown *in vitro* antibacterial and antibiotic sensitizing activity against *E. coli* AG102, which is a multidrug-resistant (MDR) gram-negative enteric bacterium, and against *P. stuartii* strains. This study observed a synergistic effect of these substances with a PA*β*N efflux pump inhibitor. The antibacterial potential was improved by 73.37% with crude MFS against the tested MDR, whereas it was improved by 100% with 3′,4′,7-trihydroxyflavone. Therefore, both substances are considered substrates for efflux pumps because they have intracellular targets [166]. There was a synergistic action between the extracts and at least one of the six antibiotics tested against 50% of MDR bacterial strains. The compound 3′,4′,7-trihydroxyflavone improved the activity of 70% of the antibiotics tested. These results suggest that this compound may be considered as a potential efflux pump inhibitor because of its antibacterial effect and antibiotic-modifying activity [166].

The effects of the hydroalcoholic extract of *Glycyrrhiza glabra* and its flavonoids were evaluated in an *in vivo* model of *P. aeruginosa*-induced pulmonary infection in rats. The study elucidated the mechanism of action, inhibition of biofilm formation, pathogenesis, and efflux activity of one of its pure glycyrrhizic acid components [167]. The findings were validated using molecular docking analysis using ExoS segmentation, which confirmed the potential of the herb *G. glabra* [153]. Isolated *G. glabra* glycosides altered membrane permeability and inhibited efflux activity and biofilm formation by *P. aeruginosa* [166]. These flavonoids isolated from licorice showed inhibitory effects on acute lipopolysaccharide-induced pneumonia [167]. These studies provide evidence of preclinical efficacy of *G. glabra* in *P. aeruginosa* pneumonia.

In addition to interfering with the QS and efflux pump, antimicrobials act by direct killing of microbial cells. Antibacterial activity was evaluated by MIC in DNA fragmentation test, caspase activity, lipid peroxidation, inner and external membrane permeabilization, membrane fluidity disturbance, and membrane damage. Isoquercitrin isolated from the perennial herb *Aster yomena*, generally found in Korea and Japan, inhibited *E. coli* growth or completely destroyed bacterial cells. Sub-MIC concentrations of isoquercitrin led to a rapid increase in DNA fragmentation and caspase activation, which are characteristics of apoptosis. The antibacterial activity of isoquercitrin in *E. coli* is attributed to membrane alterations, most likely caused by the induction of oxidative stress and apoptosis [167]. A double-blind, placebo-controlled clinical trial showed that propolis oral spray could be used to improve and immediately resolve the symptoms of uncomplicated upper respiratory tract bacterial infections, without any pharmacological treatment [168].

The antibacterial actions of flavonoids and flavonols range from QS disturbance and alterations in the efflux pump to direct induction of apoptosis (Table 4). Unfortunately, there are few studies detailing the mechanisms involved, but their microbicidal and synergistic effects with antibiotics should be further explored in the future.

## 3. Concluding Remarks

Conclusively, flavonoids are bioactive components found in fruits and vegetables being recognized as highly versatile substances with therapeutic applications, representing a vast source of pharmacological potential. Herein, we discuss the pivotal role of some flavonoids against inflammation and bacterial infection, which are responsible for millions of casualties every year and severely affect hospitalized and susceptible individuals. Currently available drugs used to treat of these individuals will probably no longer be effective shortly. Bioactive compounds derived from plants play a critical role in treating or preventing diseases either individually or synergistically with antibiotics. Furthermore, flavonoids play a critical role in modulating oxidative stress and treating inflammatory and infectious diseases, particularly those caused by resistant and opportunistic bacteria, through diverse mechanisms of action. Despite their low bioavailability, a proper delivery system such as nanoformulation may aid in their clinical applications. Nanotechnology offers multiple benefits in treating chronic human diseases by site-specific and target-oriented delivery of precise medicines, improving the efficacy of drugs and natural products [169, 170]. For instance, phytochemical cyclodextrin complexes have the potential for transformation into drug delivery systems [171], and nanotechnology-based drug delivery for therapeutics are bioactive compounds from plant sources [172]. Besides, plant phenolic compounds have potential use as a natural feed additive [173], enhancing antioxidant status, immune function, and growth performance of farm animals [174]. We focused on the reported mechanisms and intracellular targets of flavonols and flavones (Figure 6) to boost research on discovering bioactive compounds and their mechanisms of action, anticipating that they can be used as standard treatment for inflammatory and infectious diseases in the future.

## Figures and Tables

**Figure 1:** The basic skeleton of flavonoids (C6-C3-C6).

**Figure 2:** Chemical structures of some representative flavonoids and the basic skeleton of the flavonoids in the middle.

**Figure 3:** Chemical structures of quercetin, myricetin, and kaempferol.

**Figure 4:** Chemical structures of luteolin and apigenin.

**Figure 5:** Chemical structures of 3′,4′-dihydroxyflavone, baicalein, scutellarein, lucenin-2, vicenin-2, diosmetin, nobiletin, tangeretin, and 5-O-methyl-scutellarein.

**Figure 6:** Summary of the effects of flavonols and flavones. The figure presents a range of signaling pathways of the inflammatory process and the stages where the compounds block the signaling cascade. The number represents the pathways inhibited by different compounds. For example, pathway 1 is blocked by the following compounds: quercetin, luteolin, 3′,4′-dihydroxyflavone, baicalein, nobiletin, and tangeretin. Scutellarin, vicenin-2, apigenin, 5-O-methyl-scutellarin, and the substances are able to block pathway 1 and inhibit pathway 2. Only luteolin and lucenin-2 inhibit pathway 3. Furthermore, pathway 4 can only be inhibited by luteolin. Most of the compounds previously mentioned in this review block pathway 5, except nobiletin, tangeretin, vicenin-2, and lucenin-2. Furthermore, luteolin, scutellarin, vicenin-2, and lucenin-2 inhibited pathway 6. Only isoquercetin blocks pathway 7, and luteolin blocks pathway 8.

**Table 1:** Natural sources and content (mg/100 g or mg/100 ml) of some flavonols and flavones.

Substance	Food source	Estimated content (mg/100 g fresh weight)	Reference
Quercetin	Tomatoes	7-55	[26]
	Lettuce	2-911	
	Onions	10-1359	
	Peas	98-145	
	Apple	2-26	[22]
	Apricot	2-5	
	Broccoli	0-3	
	Chives	10-30	
	Cramberry	149	
	Grape, red	1-3	
	Cramberry	25	[44]
	Oregano	42	
	Dill	79	
	Lovage	170	[45]
	Radish leaves	70	
	Watercress	29	

Kaempferol	Kale	47	[44]
	Spinach	55	
	Chives	12	
	Dill	40	
	Cabbage	20-25	[45]
	Watercress	23	

Luteolin	Celery	6-40	[26]
	Mexican oregano	901-1137	[46]
	Spices, celery seed	811	[47]

Apigenin	Celery	17-191	[26]
	Spinach	1	[48]
	Green pepper	0-1	
	Welsh onion	8-11	
	Parsley	4503	[49]
	Chamomile	300-500	
	Vine-spinach	62	

Baicalein	Wine, tea, citrus fruits, dark chocolate, and herbs	n.d.	[50]
	Roots of *Scutellaria baicalensis (traditional Chinese herbal medicine)*	n.d.	[51]
	Welsh onion	9	[48]
	Spinach	19	

Scutellarein	Mexican oregano	24-48	[47]

Tangeretin	Citrus fruits, Orange juice (pure)	8∗	[52]

Nobiletin	Grape fruits, teas (*Camellia sinensis*), herbal tea, and black tea	n.d.	[53]

n.d.: not described; ^∗^mg/100 ml.

**Table 2:** Anti-inflammatory effect of flavonols.

Flavonoid	Experimental Model	Treatment/dose	Mechanism of action or main results	Author/year
Quercetin	***In vivo*** Acetic acid induced ulcer gastric in male Wistar rats	2.5, 5 and 10 mg/kg	(i)Reduction of expression of the pro-inflammatory cytokines TNF-*α* and IL-6 (ii)Inhibition of COX-2	[99]
	***In vivo*** Isoproterenol-induced myocardial infarction in Wistar rats	50 mg/kg	(i)Protection against heart damage (ii)Attenuation of oxidative stress (iii)Protection of cardiac architecture (iv)Modulation of calpain expression (v)Reduction of expression of the pro-inflammatory cytokines TNF-*α* and IL-6	[98]
	***In vitro*** Human colonic epithelial cell line Caco-2 cell	200 *μ*M	(i)Inhibition of NLRP3 activation (ii)Reduced ROS production (iii)Reduction in IL-1 and IL-18 levels	[105]
	***In vivo*** Acute necrotizing pancreatitis (ANP) model in rats	50 mg/kg	(i)Mitigation of damage to the pancreas, ileum, and intestine (ii)Suppression of TLR4/MyD88/p38 and inhibition of endoplasmic reticulum stress	[103]
	***In vitro*** Human middle ear epithelial cells (HMEECs), renal epithelial cells (HK2), and mouse lung epithelial cells (MLE-12), human liver epithelial cells (L02), and human lung epithelial cells (BEAS-2B)	40, 80 and 120 *μ*M	(i)Suppressed NTHi-induced CXCR4 expression levels *in vitro* and *in vivo* (ii)Blocked CXCR4 activation through direct IKK*β* phosphorylation inhibition	[102]
	***In vivo*** Otitis NTHi-induced in mice	20, 40 and 80 mg/kg		

Isoquercetin	***In vivo*** Streptozotocin-induced diabetes in male Wistar rats	40 mg/kg	(i)Reduction in inflammation marker levels (IL-1*β*, C-reactive protein, and MPC-1) (ii)Restoration of plasma antioxidant capacity (iii)Inhibition of 12/15-LOX activity in the lungs and liver (iv)Upregulation of HO-1 expression in the joints and lungs (v)Reversal of weight loss, reduction in glucose levels, and increase in insulin production (vi)Increased SOD and CAT activity (vii)Suppression of the inflammatory genes NF-*κ*B, IL-1, IL-6, TLR, TNF-*α*, and COX-2	[109]

Kaempferol	***In vitro*** Anti-adipogenic effects on 3 T3-L1 cells	7.5, 15, and 30 *μ*M	(i) Blockage of 3 T3-L1 differentiation and lipid accumulation in mature adipocytes (ii)Reduction in expression of the adipogenic markers PPAR*γ* and C/EBP*α* in 3 T3-L1 cells	[108]
	***In vivo*** Wild-type zebrafish	5, 10, and 20 *μ*M		
	***In vitro*** Anti-adipogenic effects on 3 T3-L1 cells	20, 40, 60, 80, 100, 120, 150, and 170 *μ*M	(i)Modulation of adipogenic gene expression in mature adipocytes (ii)Decreased accumulation of lipids in mature adipocytes (iii)Upregulation of Pnpla2 and Lipe mRNA expression	[110]

Myricetin	LPS stimulated H9c2 cells	H0, 10, 30, and 50 *μ*M	(i)Reduction in cleaved caspase-3 and Bcl-2 levels (ii)Increase in Bax levels in H9c2 cells (iii)Reduction in MCP-1/CCL-2 and I*κ*B*α* phosphorylation levels	[111]

**Table 3:** Mechanisms underlying anti-inflammatory action of flavones.

Flavonoid	Experimental Model	Treatment	Mechanism of action or main results	Author/year
Luteolin	***In vitro*** Rat chondrocytes	25, 50, and 100 *μ*M	(i)Reduction of the levels of NO, PGE2, TNF-*α*, MMP-2, MMP-8, and MMP-9 induced by IL-1*β* (ii)Reduction of the expression of COX-2, iNOS, MMP-1, MMP-3, and MMP-13 (iii)Reversal of IL-1*β*-induced collagen II degradation (iv)Inhibition of IL-1*β*-induced phosphorylation of NF-*κ*B	[113]
	***In vivo*** *Osteoarthritis in Wistar rats*	10 mg/kg	(i)Prevention of cartilage destruction and increased collagen II expression in rats	
	***In vitro*** Cardiomyocytes	5 e 10 *μ*g/kg	(i)Reduction of inflammatory mediator production (ii)Inhibition of oxidative stress (iii)Inhibition of the NF-*κ*B pathway (iv)Activation of the NRF2 pathway	[122]
	***In vivo*** Mice C57BL/6 with diabetes type I induced by streptozotocin	20 mg/kg	(i)Inhibition of fibrosis, hypertrophy, and cardiac dysfunction in streptozotocin-induced diabetic mice	
	***In vitro*** Human neutrophils	3, 10, and 30 *μ*M	(i)Inhibition of superoxide anion production (ii)Inhibition of NO production and NET formation in neutrophils (iii)Reduction in elastase production and inhibition of CD11b expression and chemotaxis (iv)Inhibition of ERK and kinase-1 activated protein (MEK-1)	[1]
	***In vivo*** Male mice (C57BL/6) Paw edema CFA-induced	50 mg/kg	(i)Reduction of neutrophil infiltration (ii)Improvement in adjuvant-induced edema (iii)Reduction in ROS production	
	***In vivo*** Swiss albino mice Paw edema carrageenan-induced	10, 25, and 50 mg/kg	(i)Reduction in the number of abdominal constrictions and licking induced by acetic acid and glutamate (ii)Inhibition of nociceptive response in both phases of formalin test (iii)Inhibition of carrageenan-induced paw edema (iv)Reduction in the levels of TNF-*α*, IL-1*β*, and IL-6	[117]
	***In vivo*** BALB/c mice Model of mastitis induced by *S. aureus*	25, 50, and 100 mg/kg	(i)Protection of tissue destruction of mammary glands (ii)Inhibition of inflammatory cell infiltration (iii)Inhibition of TNF-*α*, IL-1*β*, and IL-6 expression (iv)Inhibition of I*κ*B*α* and NF-*κ*B p65 phosphorylation levels (v)Downregulation of MMP-2 and MMP-9 expression (vi)Increase in the levels of tissue metalloproteinase inhibitors (TIMP)-1 and TIMP-2	[125]
	***In vivo*** Male BALB/c mice model of hepatic cancer chemically induced	1, 5, 10, 20 and 50 *μ*g/kg	(i)Modification in the levels of *α*-fetoprotein and antioxidant enzymes (SOD and CAT) (ii)Modification of enzymatic markers such as AST and ALT (iii)Reduction in the levels of glutathione and inflammatory cytokines such as IL-2 and IFN-*γ* in the plasma and liver	**[** 140 **]**
	***In vitro*** Colon tumor cell HT-29	50 *μ*M and 100 *μ*M	(i)Inhibition of IL-8 production, and COX-2 and iNOS expression (ii)Downregulation of the JAK/STAT signaling pathway	[123]
	***In vitro*** Primary cultures of rat cortical cells subjected to oxidative stress	3–30 *μ*M	(i)Attenuation of oxidative damage (ii)Inhibition of ROS generation (iii)Increase in bad phosphorylation in serine-112 (iv)Attenuation of induced caspase-3 activation (v)Upregulation of HO-1 expression (vi)Increase in the levels of ERK, p38, JNK, and AKT phosphorylation	[141]

Apigenin	***In vivo*** Model of bleomycin-induced lung fibrosis in Wistar rats	10, 15, and 20 mg/kg/day	(i)Prevention of pulmonary fibrosis (ii)Prevention of bleomycin-induced inflammation by decreasing TNF-*α* and TGF-*β*1 levels (iii)Attenuation of reduced SOD activity (iv)Inhibition of leukocyte infiltration	[128]

3′,4′-dihydroxyflavone	***In vitro*** Murine BV2 microglial cells	0-10 *μ*M	(i)Inhibition of the production of NO and PGE2 chemokines (ii)Inhibition of pro-inflammatory cytokines such as TNF-*α*, IL-1*β*, and IL-6 (iii)Inhibition of MAPK phosphorylation (iv)Inhibition of the NF-*κ*B pathway	[129]
	***In vivo*** Male C57BL/6 mice	5 Mg/kg	(i)Inhibition of LPS-mediated iNOS and COX-2 expression (ii)Reduces LPS-induced neuroinflammation in the mouse brain	

Baicalin	***In vivo*** Rotenone-induced brain injury in rats Sprague-Dawley (SD) rats	200 mg/kg	(i)Mitigation of motor deficit (ii)Attenuation of brain injury (iii)Suppression of the production of TNF-*α* and IL-6 (iv)Modulation of activation of astrocytes and microglia (v)Blockage of NF-*κ*B activation (vi)Inhibition of the MAPK pathway	[142]

Scutellarin	***In vitro*** (LPS)-induced cognitive deficit in male albino Wistar rats	5, 25, or 50 mg/kg/day	(i)Dose-dependently improved spatial deficit and recognition memory (ii)Decreased expression of NF-*κ*B, TNF-*α*, and IL-6	[130]

Lucenin-2 Vicenin-2	***In vitro*** Murine monocyte/macrophage cell line	0, 1, 10, and 100 mg/mL	(i)Inhibition of NO production and reduction of iNOS and COX-2 expression	[133]

Vicenin-2	***In vitro*** LPS stimulated inflammatory activities in PMA-differentiated THP-1 cells and human primary mononuclear cells	1.6-160 nM	(i)Stimulated IL-18 decrease (ii)Inhibition of the NF-*κ*B pathway—increase in P50 transcriptional subunit homodimerization	[135]

Nobiletin	***In vivo*** AP induced with L-arginine in male C57BL/6 mice	50 mg/kg	(i)Reduction in plasma amylase levels (ii)Reduction in myeloperoxidase activity in the pancreas (iii)Inhibition of inflammatory factors (iv)Inhibition of phosphorylated p38 and AKT	[136]

Tangeretin	***In vitro*** LPS-stimulated dendritic cells	5, 10, or 20 *μ*M	(i)Inhibition of TNF-*α*, IL-12, and IL-23 expression (ii)Inhibition of the NF-*κ*B and MAPK pathways (iii)Activation of myeloperoxidase activity (iv)Inhibition of Th1 and Th17 cell differentiation (v)Inhibition of T-bet and ROR*γ*t expression (vi)Inhibition of IFN-*γ*, IL-12, and IL-17	[137]
	***In vivo*** Colitis TNBS-induced in male mice C57BL/6	10 or 20 mg/kg	(i)Tangeretin may attenuate colitis by inhibiting IL-12 and TNF-*α* expression	[137]

5-O-methyl-scutellarein	***In vitro*** LPS stimulations in murine macrophages RAW 264.7 cells	2, 10, and 50 *μ*g/mL	(i)Dose-dependent inhibition of total cell recruitment (ii)Inhibition of neutrophil infiltration (iii)Reduction in the levels of TNF-*α*, IL-1*β*, and IL-10	[138]
	***In vivo*** Lipopolysaccharide (LPS) -induced peritonitis model in mice Swiss Webster	4 and 20 mg/kg	(i)Decreased leukocyte migration to the peritoneal cavity and a reduction in the concentrations of pro-inflammatory cytokines (TNF*α* and IL-1*β*)	

Diosmetin	***In vivo*** Colitis TNBS-induced	50, 100, and 200 mg/kg	(i)Showed protective effect by suppression of TNF-*α*, IL-6 and NF-*κ*B (ii)Elevation of SOD and CAT levels in the colonic mucosa and depletion of MDA which further confirms the antioxidant activity of diosmetin in ulcerative colitis	[132]

**Table 4:** Antibacterial actions of flavonoids.

Flavonoid	Experimental Model	MIC	Mechanism of action or main results	**Author/year**
3′,3′,4-trihydroxyflavone	***In vitro*** Pathogens: *E. faecalis, S. aureus*, *E. coli*, *E. aerogenes*, *S. epidermidis*, *K. pneumoniae S. haemolyticus*, and *P. aeruginosa*	32 *μ*g/mL (*E. faecalis* and *S. aureus*) 64 and 128 *μ*g/mL (*K. pneumoniae*, *E. aerogenes*, and *E. coli*)	(i)Killing bacteria from diabetic wounds	[153]

3′,4′,7-trihydroxyflavone	***In vitro*** Pathogens: *E. coli*, *E. aerogenes*, *K. pneumoniae*, *P. stuartii*, and *P. aeruginosa*	MIC values ranging from 4 to 128 *μ*g/mL	(i)Antibacterial and antibiotic sensitizing activity against MDR gram-negative enteric bacteria Substrates for efflux pump	[166]

Isoquercitrin	***In vitro*** Pathogen: *E. coli*	MIC 4.64 *μ*g/mL MBC 18.56 *μ*g/mL	Membrane alterations, a rapid increase in DNA fragmentation, and caspase activation	[167]

Baicalin	***In vitro*** Broth-microdilution method	Sub-MIC 256 *μ*g/mL	(i)Anti-QS activity against *P. aeruginosa* (ii)Marked reduction in inflammation indicated by reduced accumulation of cellular infiltration in peritoneal tissue Significant decrease in IL-4 in the peritoneal flushing fluid Significant increase in INF-*γ* production	[160]
	***In vivo*** Mouse intraperitoneal foreign-body biofilm infection model	100 mg/kg subcutaneous		

Rutin	***In vitro*** AI-2 bioluminescence assay APEC-O78 strain (CVCC141)	12.5, 25 and 50 *μ*g/mL	(i)Inhibition of QS gene expression in *P. aeruginosa* (ii)Decreased production of the signaling molecule AHL by *P. aeruginosa* (iii)Reduction in CFU count of *P. aeruginosa*	[162]
